# Sex-Specific Intubation Biomechanics: Intubation Forces Are Greater in Male Than in Female Patients, Independent of Body Weight

**DOI:** 10.7759/cureus.8749

**Published:** 2020-06-21

**Authors:** Bradley J Hindman, Franklin Dexter, Benjamin C Gadomski, Martin J Bucx

**Affiliations:** 1 Anesthesia, University of Iowa, Iowa City, USA; 2 Anesthesiology, University of Iowa, Iowa City, USA; 3 Mechanical Engineering, Colorado State University, Fort Collins, USA; 4 Anaesthesiology, Pain and Palliative Medicine, Radboud University Medical Center, Nijmegen, NLD

**Keywords:** biomechanics, cervical spine, force, gender, intubation, laryngoscopy, sex differences

## Abstract

Background

Studies of head, neck, and cervical spine morphology and tissue material properties indicate that cervical spine biomechanics differ between adult males and females. These differences result in sex-specific cervical spine kinematics and injury patterns in response to standardized loading conditions. Because direct laryngoscopy and endotracheal intubation require the application of a load to the cervical spine, intubation biomechanics should be sex-specific. The aim of this study was to determine if intubation forces during direct laryngoscopy differ between male and female patients and, if so, is the difference independent of body weight.

Methods

We pooled original data from three previously published adult clinical intubation studies that used methodologically reliable intubation force measurements (measured total laryngoscope force applied to the tongue, and force values were insensitive to or accounted for other laryngoscope blade forces). All patients had undergone direct laryngoscopy and orotracheal intubation with a Macintosh 3 blade under general anesthesia. Patient data included sex, age, height, weight, and maximum intubation force. Least squares multivariable linear regression was performed between the dependent variable (maximum intubation force) and two independent variables (patient sex and patient weight). A third term was added for the interaction between patient sex and weight.

Results

Among all patients (males n=42, females n=59), the median intubation force was 42.2 N (25^th^ to 75^th^ percentiles: 31.5 to 57.4 N). While controlling for patient body weight, intubation force differed between the sexes; P=0.011, with greater intubation force in male patients. While controlling for patient sex, there was a positive association between patient body weight and intubation force; P=0.009. In addition, there was a significant interaction between patient sex and weight; P=0.002, with intubation force in male patients having greater dependence on body weight. The difference in intubation force between male and female patients who had the same body weight exceeded 5 N when body weight exceeded 75 kg, and intubation force differences between male and female patients increased as patient body weight increased. Additional analyses using robust regression and using body mass index instead of weight provided comparable results.

Conclusion

In adult patients, the biomechanics of direct laryngoscopy and intubation are sex-specific. Our findings support the need to control for patient sex and weight in future clinical and laboratory studies of the human cervical spine and head and neck biomechanics.

## Introduction

Recent studies of head, neck, and cervical spine morphology [1-4] and tissue material properties [5-6] indicate adult male and female cervical spines are significantly different [7]. In finite element (FE) modeling studies, these differences result in sex-specific cervical spine kinematics in response to standard loads [8] and may explain sex-specific cervical spine injury patterns in response to inertial loading [9]. Direct laryngoscopy and endotracheal intubation is a common clinical procedure in which a load is applied to the cervical spine. Specifically, using a laryngoscope blade, over a few seconds the clinician applies 40-50 N force to the patient’s tongue, which simultaneously causes craniocervical extension and tongue and mandible displacement [10]. These motions create a line of sight between the maxillary incisors and the posterior glottis, enabling the clinician to insert an endotracheal tube via the mouth into the patient’s trachea under direct vision. Collectively, the aforementioned morphologic, biomechanical, and modeling studies suggest intubation biomechanics should be sex-specific.

Three clinical studies have reported intubation forces were greater in male patients [10-12], which is consistent with intubation biomechanics being sex-specific. One study made a direct male versus female patient comparison (P<0.001) [11], one study was descriptive only and did not make a formal comparison [12], and one study reported intubation force differences between direct- and video-laryngoscopy were greater in male patients (P=0.0070) [10]. In all three studies, greater intubation forces in male patients appeared to be related to their greater body weight. Because of small sample sizes, these three studies lacked statistical power to determine if intubation force differences between male and female patients were independent of body weight.

The aim of this study was to determine if intubation forces during direct laryngoscopy differ between male and female patients and, if so, is the difference independent of their body weight. To increase statistical power, the authors pooled data from previously published clinical intubation studies that were selected on the basis of their methodological reliability.

## Materials and methods

Literature search and study selection

On December 7, 2019, one author (BH) conducted a PubMed search to identify clinical intubation studies reporting quantitative values for intubation force. Search criteria are summarized in Table 1, yielding 340 citations.

**Table 1:** PubMed search criteria MeSH: Medical Subject Heading

Criteria	Terms	Citations, n
1. MeSH term	Laryngoscope OR laryngoscopy OR intubation, endotracheal	44,064
2. Text in title OR abstract	Force OR forces	320,571
3. 1 AND 2		340

After reading abstracts and/or full text, 323 citations were excluded because laryngoscope force measurements were: (1) not reported (n=275); (2) obtained only from manikins, cadavers, or other models (n=34); (3) qualitative, not quantitative (n=7); 4) limited to forces applied to maxillary incisors (n=4); 5) experimentally fixed, not variable (n=2); or 6) obtained in children (n=1) (complete search results are available from the corresponding author upon request).

Among the remaining 17 adult intubation force studies, two studies reanalyzed data originating from a preceding or companion paper, leaving 15 primary adult intubation force studies. Among the 15 studies, almost all used a unique method/device to measure intubation force. Within an individual study, device-related force measurement errors will be comparable among patients, allowing for comparisons within the study. However, in order to pool data among studies, intubation force values from different studies must have comparable accuracy. To make accurate intubation force measurements, devices must: (1) measure laryngoscope contact forces applied to the entire surface of the tongue; (2) be insensitive to or account for the spatial distribution (or application point) of forces applied to the tongue; and (3) be insensitive to or account for laryngoscope blade forces applied to other structures such as the maxillary incisors. Among the 15 primary adult intubation force studies, three studies used methods that satisfied these methodologic criteria (a complete discussion is available from the corresponding author upon request ). In brief, two studies by Bucx et al. utilized force and moment sensors in the laryngoscope handle and accounted for laryngoscope blade forces applied to maxillary incisors [13-14]. The study by Hindman et al. used a thin multisensor force mat covering the entire laryngoscope blade contact surface that was insensitive to force applied to maxillary incisors [10]. Intubation force values were very similar among these three studies. The two principal investigators of these three studies agreed to share data for this new analysis.

Clinical study methods

The University of Iowa Institutional Review Board (IRB) determined that this study does not meet the regulatory definition of human subjects research because it is an analysis of de-identified data (IRB 202001091, January 13, 2020). Consequently, individual patient consent was not required.

Original data from two previous clinical studies were provided by an author (MB) [13-14]. Both studies were conducted at Erasmus University, Rotterdam, The Netherlands, had been approved by the Hospital Ethics Committee, and written informed consent was obtained from all patients. These two studies were conducted between 1992 and 1994, predating clinical trial registration databases. In the first study, all patients were intubated using a Macintosh 3 blade [13]. In the second study, patients were randomized to be intubated with either a conventional or modified Macintosh 3 blade [14]. Only conventional Macintosh 3 intubation force data were used in this analysis. Additional original data from a previous randomized clinical trial were provided by author BH [10]. The study had been approved by the University of Iowa Institutional Review Board (IRB 201102721) and written informed consent was obtained from all patients. The study was registered prior to patient enrollment at www.ClinicalTrials.gov (NCT01369381, Principal investigator: Bradley J. Hindman, date of registration: June 8, 2011). Patients were intubated twice in random order, once utilizing direct laryngoscopy with a Macintosh 3 blade and once utilizing a videolaryngoscope. Only Macintosh 3 intubation force data were used in this analysis.

In all three studies patients were selected on the basis that easy intubation was expected. Airway morphology was characterized in one study [10]. All laryngoscopists were non-trainees; years of postgraduate experience was reported in one study [10]. All patients underwent direct laryngoscopy and orotracheal intubation under general anesthesia after the intravenous (IV) administration of nondepolarizing neuromuscular blocking drugs. All patients were intubated on the first attempt. Intubation difficulty was characterized in one study [13]. In all studies, the glottic view was characterized using the Cormack and Lehane scale [15].

Statistical analysis

Study data were provided without patient identifiers: patient sex, age, height, weight, and both maximum and mean intubation force. Data from the three studies were pooled for analysis. Because (1) maximum cervical spine motion during laryngoscopy is related to maximum laryngoscope force application [10] and (2) cervical spinal cord strain is related to laryngoscope force application [16], maximum intubation force was selected a priori as the outcome (dependent) variable. Least squares multivariable linear regression was performed between this dependent variable and two independent variables: patient sex and patient weight. A third term was added for the interaction between patient sex and weight. In this model, the residual versus the fitted plot did not show significant heteroscedasticity (Breusch-Pagan/Cook-Weisberg test P=0.0657). However, because there was a tendency toward heteroscedasticity and several marked outlier values were present, a second analysis was performed using STATA (StataCorp, College Station, Texas) robust regression, which is less sensitive to outliers than the conventional methods. Calculations were performed using STATA 16.0 functions (in sequence): summarize, regress, hettest, and rreg. As a secondary analysis, the same analysis methods were used with body mass index (BMI; weight/(height)^2^) rather than body weight as an independent variable. All P-values were two-sided, with the threshold for significance equal to 0.05.

The sample size was unchangeable because this is a historical cohort study. To evaluate whether our sample size was sufficiently large for results to be reported, we considered a difference in the marginal effect of patient sex on maximum intubation force of 5 N (10% of the median maximum value) to be potentially clinically important. The marginal effect of patient sex was estimated using the STATA margins function.

## Results

Patient characteristics, intubation characteristics, and maximum intubation forces are summarized in Table 2. Intubation force values were comparable among the three studies. Among all patients, the median intubation force was 42.2 N (25th to 75th percentiles: 31.5 to 57.4 N). Among male (n=42) and female patients (n=59), weight overlapped between 55 and 95 kg (males n=37, females n=52).

**Table 2:** Patient characteristics, intubation characteristics, and intubation forces Values are reported as number, percentage, or median (25th to 75th percentiles). *One female patient missing height and body mass index data. †Cormack and Lehane glottic visualization scale [15]. 1: Most of the glottis visible. 2: Only the posterior aspect of the glottis visible (at least the arytenoids). 3: No part of the glottis seen, but epiglottis seen. 4: Not even the epiglottis seen. ‡Originally reported as Percentage of Glottic Opening (POGO): 74±16% (mean ± SD). 12/14 patients had POGO ≥60%, equivalent to Cormack and Lehane grade 1. 2/14 patients had POGO scores of 40% and 50%, equivalent to grade 2.

	Bucx et al., 1994 [13]	Bucx et al., 1997 [14]	Hindman et al., 2014[10]	Pooled
Patients	65	22	14	101
Sex, female	37 (57%)	13 (59%)	9 (64%)	59 (58%)
Age, years	51 (39 to 60)	53 (35 to 65)	49 (25 to 65)	51 (38 to 61)
Weight, kg	67 (60 to 80)	75 (58 to 82)	72.5 (65.0 to 85.7)	70 (60 to 82)
Body mass index, kg/m^2 ^	24.2 (21.7 to 27.6)^*^	23.7 (22.2 to 26.2)	27.2 (23.7 to 28.5)	24.2 (21.8 to 27.7)^*^
Laryngoscopists	12	5	2	19
Glottic view†				
Grade 1	61 (94%)	19 (86%)	12 (86%)^‡^	92 (91%)
Grade 2	4 (6%)	2 (9%)	2 (14%)	8 (8%)
Grade 3	0	1 (5%)	0	1 (1%)
Maximum intubation force, N	40.3 (31.4 to 53.0)	47.5 (33.2 to 57.4)	48.4 (37.6 to 65.8)	42.2 (31.5 to 57.4)

Primary analysis results are summarized in Table 3 and shown graphically in Figures 1A-1B.

**Table 3:** Primary analysis models using the maximum intubation force as the dependent variable and patient sex and weight as independent variables Values are reported as the parameter estimate (standard error of the estimate), P-value. Positive values for the parameter estimates for patient sex indicate a greater maximum intubation force for male patients.

Primary Analysis Model	Patient Sex	Patient Weight	Sex/Weight Interaction
Multivariable least-squares linear regression	55.68 (21.35), P=0.011	0.54 (0.20), P=0.009	-0.90 (0.29), P=0.002
Robust regression	37.97 (17.33), P=0.031	0.47 (0.17), P=0.006	-0.67 (0.23), P=0.005

**Figure 1:** Patient weight, sex, and maximum intubation force A) Individual values for patient weight (kg) and maximum intubation force (N) in females (blue circles) and males (red diamonds) with corresponding linear regression lines for females (blue; slope = -0.36; 97.5% confidence interval -0.82 to 0.10) and males (red; slope=0.54; 97.5% confidence interval 0.08 to 1.00). B) Conditional marginal effects of patient sex as a function of patient weight. Positive values indicate a greater intubation force in male patients. Error bars show 95% confidence interval.

In both primary analysis models (i.e., least-squares regression and robust regression), while controlling for patient body weight, intubation force significantly differed between male and female patients; P=0.011 and P=0.031, respectively, with a greater maximum intubation force in male patients. In both primary models, while controlling for patient sex, there was a significant positive association between patient body weight and maximum intubation force, P=0.009 and P=0.006, respectively. In both primary models, there was a significant interaction between patient sex and weight; P=0.002 and P=0.005, respectively. As shown in Figure 1B, as patients’ body weight increased, intubation force differences between male and female patients progressively increased, with differences exceeding 5 N when patients’ weight exceeded 75 kg.

Secondary analysis results are summarized in Table 4 and shown graphically in Figures 2A-2B.

**Table 4:** Secondary analysis models using maximum intubation force as the dependent variable and patient sex and body mass index (BMI) as independent variables Values are reported as the parameter estimate (standard error of the estimate), P-value. Positive values for the parameter estimates for patient sex indicates a greater maximum intubation force for male patients.

Secondary analysis model	Patient Sex	Patient BMI	Sex/BMI Interaction
Multivariable least-squares linear regression	54.39 (25.28), P=0.034	1.91 (0.75), P=0.012	-2.61 (1.00), P=0.011
Robust regression	41.19 (20.43), P=0.047	1.60 (0.61), P=0.010	-2.14 (0.81), P=0.010

**Figure 2:** Patient body mass index (BMI), sex, and maximum intubation force A) Individual values for patient BMI (kg/m^2^) and maximum intubation force (N) in females (blue circles) and males (red diamonds) with corresponding linear regression lines for females (blue; slope = -0.69; 97.5% confidence interval -2.21 to 0.82) and males (red; slope=1.91; 97.5% confidence interval 0.20 to 3.62). B) Conditional marginal effects of patient sex as a function of patient body mass index (BMI). Positive values indicate a greater intubation force in male patients. Error bars show a 95% confidence interval.

In both secondary analysis models, while controlling for patient BMI, intubation force significantly differed between male and female patients; P=0.034 and P=0.047, respectively, with a greater maximum intubation force in male patients. In both secondary models, while controlling for patient sex, there was a significant positive association between patient BMI and maximum intubation force; P=0.012 and P=0.010, respectively. In both secondary models, there was a significant interaction between patient sex and BMI; P=0.011 and P=0.010, respectively. As shown in Figure 2B, as patients' BMI increased, the differences in intubation force between male and female patients progressively increased, with differences exceeding 5 N when patients’ BMI exceeded 26 kg/m^2^.

## Discussion

In this historical cohort study, we pooled data from three prior clinical intubation studies. We observed intubation forces differed between male and female patients, independent of their body weight. This demonstrates what might be expected but has not previously been established: intubation biomechanics are sex-specific. Based on our findings, we suggest that future clinical studies of cervical spine and head and neck biomechanics should account for both patient sex and body weight. Likewise, in FE models of the cervical spine and head and neck, sex-specific morphology and tissue biomechanical properties should be utilized whenever possible.

Sex-specific intubation biomechanics

During direct laryngoscopy displacement of airway tissue (primarily the tongue and mandible) and craniocervical spine extension are both necessary to create a line of sight between the maxillary incisors and glottis. Based on Newton’s second law of motion (force = mass x acceleration), the force required to produce these motions must be determined, at least in part, by the mass (weight) of the head, neck (cervical spine and musculature), and tongue. Our observation of greater intubation force in male than in female patients who had the same body weight suggests some or all of these structures are larger in males independent of body weight. Several studies indicate this is so. Liégeois et al. observed tongue volume was greater in males than in females, independent of either body weight or body mass index [17]. Vasavada et al. observed neck circumference was greater in males than in females independent of body weight [3], indicating a greater volume (mass) of cervical muscle, bone, and/or soft tissue in males. In a subsequent study by this group, total neck muscle volume was found to be greater in males than in females, independent of either BMI or neck circumference [4]. Stemper et al. observed that, relative to the size of the head (head circumference), cervical vertebrae were significantly larger in males [1-2]. Similarly, Vasavada et al. observed in stature- and neck-length-matched subjects that cervical vertebral dimensions were significantly larger in males [3]. Thus, the size (mass) of many anatomic structures determining intubation forces are larger in males, even when adjusted for various measures of body size, including total body weight. The expected consequence is that greater force should be required to create motion in these structures during intubation in male patients.

In addition to differences in size (mass), there are sex-specific functional differences in cervical spine biomechanics. In cadaver studies, some but not all cervical spinal ligaments show greater laxity in females [5-6]. Consequent to their smaller size, female cervical vertebrae have smaller intersegmental contact areas as compared to males, which is predicted to result in less intrinsic stability and greater motion in response to force [1-2]. Indeed, John et al. demonstrated segmental spinal motion is significantly influenced by variations in vertebral body size, specifically vertebral body depth [9]. Consistent with these observations and predictions, some [18-19] but not all [20] studies report the range of voluntary cervical spine motion is greater in females than males, even though voluntary neck muscle strength is significantly less in females [3,21]. Collectively, these morphologic and functional studies indicate the male adult cervical spine has a significantly greater stiffness than that of the female. Based on these observations, it would be expected that during intubation, male patients should require more force to create equivalent degrees of cervical spine extension.

The difference in intubation force between male and female patients progressively increased with increasing patient body weight, see Figures 1A-1B. Intubation force in male patients appeared to have a greater dependence on body weight than was observed in females. As shown in Figures 2A-2B, a very similar pattern was present in the relationship between BMI and intubation force. This observation suggests that as total body weight and/or BMI (relative adiposity) increases, the size (volume or mass) of the head, neck, and/or tongue may increase more in males than in females. This is consistent with the observation that the association between BMI and obstructive sleep apnea is stronger in males [22] and, with a given increase in weight, males have a greater increase in sleep-disordered breathing than females [23]. These differences may be due, at least in part, to sex-specific differences in the distribution of body fat, with males having a greater proportion of body fat associated with the neck [24-25].

Finite element models of the human cervical spine, head, and neck

Although FE modeling studies have provided valuable insights into spinal behaviors that otherwise would be unknown, FE models have been limited in their predictive abilities and direct clinical application. At least in part, this is because the development of traditional FE models is very time-consuming, taking months or years to produce a single spinal model. Most FE models are derived from computed tomography (CT) scans of single subjects (either male or female) and resulting FE models are assumed to be representative of the population mean. Predictions made using FE models have historically been applied to males and females with no regard for anatomical differences between sexes.

Advances in computational power have expedited the FE model development process, and patient-specific FE models have emerged that incorporate the unique anatomical features of each patient [9,26-28]. In principle, patient-specific models will account for sex-specific morphological differences. However, establishing sex-specific tissue material properties [5-6] and properly validating patient-specific FE models is an ongoing challenge. The findings of our study suggest that future studies using FE models should minimize simplifications in sex-specific differences in both anatomy and tissue biomechanical properties. In addition, FE models of cervical spine motion in response to external loading may have greater accuracy if they include cervical musculature and soft tissue structures and properties.

Limitations

A limitation of our study is that it included few obese patients. Among male and female patients, the greatest values for weight were 113 and 95 kg, respectively, and the greatest values for BMI were 35.0 and 31.3 kg/m^2^, respectively. Our study cannot predict whether sex-specific differences in intubation force would be present in patients with greater weights or BMIs. Another limitation of this study is that it does not include patients who were difficult to intubate. Because clinicians increase applied force when glottic visualization is less favorable [29-30], greater intubation forces would be expected in the setting of difficult intubation, irrespective of patient sex. In addition, our study pertains only to conventional direct laryngoscopy with a Macintosh 3 blade. Both absolute values and sex-specific differences in intubation forces may differ from those reported in this study when patients undergo intubation with different direct laryngoscope blades and/or with laryngoscopes that do not require direct line of sight, i.e., videolaryngoscopes [10].

Another limitation of our study is that it utilized data from only three of 15 primary adult intubation force studies. Pooling data from multiple studies requires data from each study to be reliable and comparable to the data from the other studies. The force measurement methods used in the three studies pooled for this analysis were methodologically reliable, quantitatively accurate, and provided nearly identical maximum intubation force values. The 12 primary studies not included in this analysis used a variety of methods to measure intubation force that resulted in variable errors, either underestimating (n=11) or overestimating intubation force (n=1) (a complete discussion is available from the corresponding author upon request). The only way these 12 other studies could have been used in this analysis is for the original force values to have been mathematically “corrected” relative to a reference value, which would necessarily have been based on the three studies used in this analysis.

## Conclusions

Our study demonstrates that intubation force (intubation biomechanics) depends on both patient sex and weight. Although sex-specific biomechanical differences are not modifiable, our findings support the need to control for patient sex and weight in future clinical and laboratory studies of the human cervical spine and head and neck biomechanics. So doing may facilitate the development of models, preventive measures, and/or spine or airway management methods to minimize cervical cord injury.
